# Deep Learning Algorithm-Based Magnetic Resonance Imaging Feature-Guided Serum Bile Acid Profile and Perinatal Outcomes in Intrahepatic Cholestasis of Pregnancy

**DOI:** 10.1155/2022/8081673

**Published:** 2022-06-06

**Authors:** Hongxue Liu, Haidong Wang, Muling Zhang

**Affiliations:** Department of Obstetrics, The Affiliated Huaian No. 1 People's Hospital of Nanjing Medical University, Huai'an, 223300 Jiangsu, China

## Abstract

This study was aimed to explore magnetic resonance imaging (MRI) based on deep learning belief network model in evaluating serum bile acid profile and adverse perinatal outcomes of intrahepatic cholestasis of pregnancy (ICP) patients. Fifty ICP pregnant women diagnosed in hospital were selected as the experimental group, 50 healthy pregnant women as the blank group, and 50 patients with cholelithiasis as the gallstone group. Deep learning belief network (DLBN) was built by stacking multiple restricted Boltzmann machines, which was compared with the recognition rate of convolutional neural network (CNN) and support vector machine (SVM), to determine the error rate of different recognition methods on the test set. It was found that the error rate of deep learning belief network (7.68%) was substantially lower than that of CNN (21.34%) and SVM (22.41%) (*P* < 0.05). The levels of glycoursodeoxycholic acid (GUDCA), glycochenodeoxycholic acid (GCDCA), and glycocholic acid (GCA) in the experimental group were dramatically superior to those in the blank group (*P* < 0.05). Both the experimental group and the blank group had notable clustering of serum bile acid profile, and the experimental group and the gallstone group could be better distinguished. In addition, the incidence of amniotic fluid contamination, asphyxia, and premature perinatal infants in the experimental group was dramatically superior to that in the blank group (*P* < 0.05). The deep learning confidence model had a low error rate, which can effectively extract the features of liver MRI images. In summary, the serum characteristic bile acid profiles of ICP were glycoursodeoxycholic acid, glycochenodeoxycholic acid, and glycocholic acid, which had a positive effect on clinical diagnosis. The toxic effects of high concentrations of serum bile acids were the main cause of adverse perinatal outcomes and sudden death.

## 1. Introduction

Intrahepatic cholestasis of pregnancy (ICP) means that most pregnant women have hepatic cholestasis in the second and third trimester of pregnancy [1–3]. It is estimated that the incidence of intrahepatic cholestasis of pregnancy in different people is between 0.3% and 15% and most reports are between 0.3% and 0.5% [4–6]. Palmer et al. [7] pointed out that the serum total bile acid level was related to the pregnancy outcome. Studies have pointed out that pregnant women with intrahepatic cholestasis of pregnancy have a unique profile of serum bile acid metabolism and hepatobiliary diseases such as hepatitis, cirrhosis, and cholelithiasis all show an increase in serum total bile acid levels, but their respective bile acid profiles are different from those of pregnant women with intrahepatic cholestasis of pregnancy [8–10]. Therefore, among pregnant women with abnormal liver function, early and accurate identification of pregnant women with intrahepatic cholestasis of pregnancy is conducive to early selection of appropriate intervention treatment and improvement of perinatal adverse outcomes.

Magnetic resonance imaging (MRI) has the characteristics of strong tissue contrast, no radiation, and strong repeatability and plays an important role in the diagnosis of liver diseases. Medical image diagnosis mainly depends on doctors' professional knowledge and clinical experience, and subjective factors may lead to different diagnosis results. As an important branch of artificial intelligence, deep learning is widely used in medical imaging [11]. The deep learning confidence network model method can automatically extract target features from massive MRI medical image data; accurately segment and identify liver anatomical structure; divide image signals of various hepatic lobes, segments, porta hepatis, hepatic arteries, portal veins, and branches of hepatic veins; establish different layers of information; and reorganize them, thus eliminating the influence of subjective factors and extracting more advanced target features, which is helpful for doctors to accurately diagnose diseases [12].

The innovation of this research was that a new MRI based on deep learning confidence network model was proposed to evaluate the imaging data of 50 pregnant women with ICP. Ultra-performance liquid chromatography-mass spectrometry/mass spectrometry (UPLC-MS/MS) was used to analyze the serum bile acid profile of ICP pregnant women in middle and late pregnancy. Then, partial least squares discriminant analysis (PLS-DA) was adopted to establish ICP diagnostic model, and the perinatal outcomes of ICP pregnant women were analyzed. This research was developed to screen differential bile acids and analyze the related factors affecting perinatal outcomes, so as to provide evidence for clinical diagnosis and treatment.

## 2. Research Methods

### 2.1. Research Objects

Fifty pregnant women with ICP diagnosed in hospital from October 15, 2019, to April 25, 2021, were selected as the experimental group. Another 50 healthy pregnant women were recruited as a blank group, and 50 patients with cholelithiasis were taken as cholelithiasis group. The age range is 24-43 years old, with an average age of (28.82 ± 5.74) years; the gestational age was 26-38 weeks at the time of enrollment. The experiment had been approved by the committee of hospital. Patients and their families understood the research situation and signed informed consent.

The inclusion criteria are as follows: (i) patients who met the diagnostic criteria for ICP in the *Intrahepatic Cholestasis Diagnosis and Treatment Expert Consensus* formulated by the expert committee for the diagnosis and treatment of intrahepatic cholestasis; (ii) ICP diagnosed at more than 28 weeks of gestation; and (iii) single fetus.

The exclusion criteria are as follows: (i) patients complicated with viral hepatitis, hepatolithiasis, acute fatty liver during pregnancy, gestational hypertension, gestational diabetes, premature rupture of membranes, placenta previa, and other diseases; (ii) patients with abnormal liver function and bile metabolism before pregnancy; and (iii) pregnant women who had congenital heart disease and other serious congenital diseases that may affect pregnancy.

### 2.2. Observation Indexes

Determinations were performed by circulating enzyme method, including fasting venous blood bile acid (TBA), total bilirubin (TBIL), conjugated bilirubin (DBIL), alanine aminotransferase (ALT), and aspartate aminotransferase (AST) of pregnant women in the experimental group and the blank group. The perinatal cord blood bile acid (TBA), creatine kinase (CK), lactate dehydrogenase (LDH) levels, cardiac troponin I (cTnI), and adverse outcomes in the experimental group and the control group were determined.

### 2.3. MRI Scan

Images were captured using 3.0 T magnetic resonance imaging and all-digital Ingenia 3.0 T superconducting magnetic resonance imaging. Liver scan was performed with 16-channel body coil, including MRI plain scan and enhanced scan. TR = 3.2 ms, TE = 1.5 ms, and reverse angle = 150. Matrix was 320 × 256, layer thickness was 3 mm, no-spacing scanning, and scanning field (FOV) = 40 cm × 32 cm. Enhanced scanning was performed with a high pressure syringe at a flow rate of 2.5 mL/s by injecting the contrast agent gadolinium penate meglumine 0.1 mmol/kg through the cubital vein mass. Then, 20 mL of normal saline was injected at a flow rate of 2.5 mL/s. The arterial phase, the portal vein phase, and the equilibrium phase were performed at 60s and 50s, respectively, 25 s after the contrast agent was injected. The serial images of all pregnant women were copied by the secondary operating station and PACs system and exported in DICOM format and stored in the mobile hard disk, and the name and number of each pregnant woman were standardized.

### 2.4. Construction of Deep Learning Belief Network Model

Restricted Boltzmann machine (RBM) is a random network model based on probability with a two-layer structure. It can meet the full connection between the layers and the disconnection within the layers and accurately improve the target characteristics. It can also be used to pre-train the traditional feedforward neural network, which greatly improves the discriminative ability of the network. If multiple RBMs are stacked, a deep learning belief network (DLBN) can be formed. Each low-level RBM is used as the input data and output after training. It is also used as the input of the high-level RBM and passed layer by layer, stacking multiple RBMs. In this way, a complete deep learning belief network structure is formed, and an abstract and characterizing feature vector is formed at the highest level (Figure 1).

### 2.5. Deep Learning Belief Network Model Training Process

The training process of deep learning confidence network model is mainly divided into the following two steps. In the pretraining stage, unsupervised layer-by-layer greedy training method is adopted. The parameters of each layer of restricted Boltzmann machine is trained from the bottom to the top. It is ensured that feature information is retained as much as possible when the low-level feature vectors are mapped to the high-level feature space. After pretraining, there is a supervised fine-tuning phase, where the parameters of each layer are fine-tuned from the top layer to the bottom layer of the network. Parameter settings include number, location, size, shape, edge blur, and neighboring organization. Combined with the characteristics of different sequences of pregnant women, the training set was trained and adjusted to obtain a complete training data set of pregnant women. In the network training process, the performance of the network will be greatly reduced if only pretraining is carried out without fine-tuning parameters. The fine-tuning process is a supervised process. It takes the difference between the output label of the network and the sample label as an error and spreads it forward layer by layer, which then modifies the parameters of each layer to make the network reach a better state, as illustrated in Figure 2.

### 2.6. Experiment Procedure

The network structure of deep learning confidence network model was built with three layers, and the last layer was connected with nonlinear classifier. MRI images were taken as training samples, and if no fine-tuning measures were taken after input into the network, the classification error rate was 21.32%. After pretraining, this was followed by supervised fine-tuning of the network to allow errors to propagate forward while adjusting parameters at each layer. The MRI test images were then fed into the adjusted network as input data. The error rate of learning classification was 5.14%, and the accuracy was increased by 16.18% compared with before fine tuning.

### 2.7. Chromatography and Mass Spectrometry Conditions

For the ACQUITY UPLC BEH C18 (50 × 2.1 mm, 1.7 *μ*m) column, the mobile phase of phase A was a 0.1% formic acid aqueous solution, and the phase B was a 0.1% formic acid-acetonitrile solution. The flow rate was 0.4 mL/min, and the column temperature was 45 °C. The gradient elution program was 0~2.5 min, 36%~45%, phase B; 2.5~3.5 min, 45%~47%, phase B; 3.5~4.5min, 47%~58%, phase B; 4.5~6.5 min, 58%, phase B; 6.5~8.5 min, 58%~65%, phase B; 8.5~10.5 min, 65%~95%, phase B; and 10.5 ~11.5 min, 36%, phase B. The electrospray ion source was in negative ion mode and multireaction monitoring mode. The capillary voltage was set to 3.5 kV, and the ion source temperature was set to 140 °C. The desolventizing gas temperature was set to 400 °C, the desolventizing gas flow rate was set to 800 L/h, and the cone gas flow rate was set to 50 L/h.

### 2.8. Statistical Methods

SPSS 21.0 was used for statistical analysis of the data. Partial least squares discriminant analysis (PLS-DA) was used to compare serum bile acid profile and screen differential bile acid spectrum among groups by using SIMCA-P 13.0 (Umetrics, Sweden). The analysis results were illustrated by two-dimensional and three-dimensional score charts. The calculated data conforming to the normal distribution were expressed as the mean standard deviation ($\overset{¯}{\text{x}}$±s), and the data that do not conform to the normal distribution is expressed as the percentage (%). In addition, *P* < 0.05 indicated notable difference.

## 3. Results

### 3.1. Experimental Results of Deep Learning Belief Network Model

The deep learning belief network model of this experiment was compared with the recognition rate of convolutional neural network (CNN) and support vector machine (SVM), and the error rate of different recognition methods on the test set was measured. The error rate of the constructed deep learning belief network (7.68%) was substantially lower than that of the convolutional neural network (21.34%) and the support vector machine (22.41%), and the difference was notable (*P* < 0.05) (Figure 3).

### 3.2. MRI Manifestations of ICP Pregnant Women

In pregnant women with ICP, the bile ducts were dilated with cholestasis, the intrahepatic bile ducts were slightly compressed by the neck of the gallbladder, and the gallbladder was retained and expanded. There was a small amount of fluid in the gallbladder fossa, and the greater omentum was wrapped in the dilated bile ducts on T2WI, showing obvious high signal, with low signal on DWI (Figures 4(a) and 4(b)). The bile duct was not dilated with biliary mud deposition, and irregular hyposignal areas were observed in the dilated bile duct with high signal intensity on T2WI, with obviously hypersignal intensity on T1WI and DWI (Figures 4(c) and 4(d)).

### 3.3. Analysis of Serum Total Bile Acid Profile in each Group

Determination of ten kinds of clear bile acids in serum of each group was carried out, including lithocholic acid (LCA), ursodeoxycholic acid (UDCA), chenodeoxycholic acid (CDCA), deoxycholic acid (DCA), cholic acid (CA), taurine lithocholic acid (TLCA), glycoursodeoxycholic acid (GUDCA), glycochenodeoxycholic acid (GCDCA), glycodeoxycholic acid (GDCA), and glycocholic acid (GCA).  Figure 5 showed ten serum bile acid profile analyses. There were different performance characteristics of serum bile acid profile in the normal healthy blank group, gallstone group, and ICP experimental group. The levels of glycoursodeoxycholic acid (GUDCA), glycochenodeoxycholic acid (GCDCA), and glycocholic acid (GCA) in the experimental group were dramatically superior to those in the blank group, and the difference was notable (*P* < 0.05). The level of glycodeoxycholic acid (GDCA) in the gallstone group was dramatically superior to that of the blank group and the experimental group, and the difference was notable (*P* < 0.05).

### 3.4. Analysis of Total Serum Bile Acid Profile between Experimental Group and Gallstone Group

According to the levels of ten known serum bile acids detected by mass spectrometry, the serum bile acid profile of the experimental group and the gallstone group was analyzed by PLS-DA, and the serum differential bile acids were screened and analyzed. The contribution values of various bile acids were the contribution values of different groups on the PLS-DA score chart. It is generally believed that bile acids with contribution values >1 are regarded as the differential bile acids between groups. The PLS-DA model (R^2^Y = 0.125, Q^2^ = 0.134) established by the experimental group and the blank group showed low values of R^2^Y and Q^2^. In Figures 6(a) and 6(b), 2D and 3D scores showed notable aggregation in both the experimental group and the blank group, and the experimental group could be well distinguished from the gallstone group.  Figure 6(c) showed that bile acids with contribution values >1 for the four differential bile acids can be used as serum differential bile acids between groups. In terms of the different bile acid contribution values of the four serums, LCA > UDCA > CDCA > DCA.

### 3.5. Analysis of Total Serum Bile Acid Profile of Experimental Group and Gallstone Group

PLS-DA scores of ten serum bile acids in the experimental group and the cholelithiasis group were established (R^2^Y = 0.258, Q^2^ = 0.195), as illustrated in Figures 7(a) and 7(b), and the serum differential bile acid spectrum was screened and analyzed. Figures 7(a) and 7(b) showed partial overlap between the experimental group and the gallstone group, indicating that the characteristics of serum bile acid profile in the two groups were similar, but there were differences in their serum bile acids.  Figure 7(c) showed that the three bile acids with contribution value >1 could be used as serum differential bile acids between groups. The bile acid contribution value of LCA was greater than UDCA and greater than CDCA.

### 3.6. Comparison of the Blood Biochemical Index Levels of Pregnant Women in the Experimental Group and the Blank Group

The levels of TBA, TBIL, DBIL, ALT, and AST of pregnant women in the experimental group were superior to those in the blank group, with notable differences (*P* < 0.05), as illustrated in Figure 8.

### 3.7. The Expression of Umbilical Cord Blood Indexes in Perinatal Infants

The comparison of the perinatal serum biochemical indexes TBA, myocardial enzyme spectrum CK, LDH, and cTnI levels between the experimental group and the blank group showed that the experimental group was dramatically superior to the blank group (*P* < 0.05), as illustrated in Figure 9.

### 3.8. Comparison of Perinatal Outcomes

Figure 10 showed the comparison of perinatal outcomes between the experimental group and the blank group. The incidence of amniotic fluid contamination, asphyxia, and premature perinatal infants in the experimental group was dramatically superior to that in the blank group, with statistical differences (*P* < 0.05).

## 4. Discussion

Intrahepatic cholestasis during pregnancy is a common clinical hepatobiliary disease that leads to adverse fetal outcomes and may lead to unexpected and sudden fetal death. Therefore, once the disease is diagnosed, intervention measures should be taken immediately [13]. Currently, for pregnant women with a gestation cycle of about 29 weeks, the measured TBA is used as an indicator of liver function, and intrahepatic cholestasis during pregnancy is screened according to whether the clinical symptoms contain pruritus [14–16]. However, the use of TBA alone as a laboratory indicator still has some limitations. Cifci et al. [17] reported that abnormal liver function occurs under normal TBA level, which cannot exclude the risk of ICP.

Serum bile acid metabolism profile of ICP pregnant women is specific. In this study, the levels of ursodeoxycholic acid, ursodeoxycholic acid, and ursodeoxycholic acid were remarkably increased in ICP pregnant women. When intrahepatic cholestasis occurs during pregnancy, liver function is impaired and bile acid concentration changes, and the levels of total bile acid and bile acid are mainly measured in clinical laboratories [18]. The results showed that the total bile acid profile of healthy pregnant women in blank group, ICP experimental group, and cholelithiasis control group was different under the premise that the total bile acid levels were similar. Therefore, serum bile acid profile had a positive effect on the clinical diagnosis of ICP, which was similar to the results of Chappell et al. [19].

ICP can cause great harm to both pregnant women and fetuses, especially the fetus [20]. The concentration of total bile acid in umbilical cord blood serum of ICP fetus will be remarkably increased, mainly due to the limitation of the process of total bile acid in the fetus to the mother. The fetus will be accompanied by hypoxia. Generally, myocardial cells are sensitive to fetal hypoxia. CK and LDH are used as specific indicators. ICP and acute hypoxia of the placenta are the direct causes of damage to the fetus. In this study, the results showed that the levels of TBA, TBIL, DBIL, ALT, AST, myocardial zymogram CK, LDH, and cTnI in the experimental group were superior to those in the control group (*P* < 0.05). The incidence of amniotic fluid contamination, asphyxia, and premature perinatal infants in the experimental group was dramatically superior to that in the blank group (*P* < 0.05). High concentrations of TBA have a direct toxic effect on the fetus, especially myocardial cells, which is the main cause of adverse perinatal outcomes and sudden death.

Starting from the research background and development of deep learning, this research studied the RBM-based deep learning model and its application in MRI. Firstly, it explained in detail how the RBM model constitutes the deep learning confidence model, and discussed the error rate of different models in the simulation experiment. Good results were harvested in the experiment, indicating that the deep learning confidence model is the optimal one [20].

## 5. Conclusion

In this research, imaging data of 50 ICP pregnant women were evaluated by constructing MRI based on deep learning confidence network model. A comprehensive analysis of serum bile acid profile in ICP pregnant women was conducted to screen for differential bile acids and to analyze perinatal outcomes in ICP pregnant women. It turned out that the error rate of deep learning confidence model was low. The serum characteristic bile acids of ICP were glycoursodeoxycholic acid, glycochenodeoxycholic acid, and glycocholic acid, which played a positive role in clinical diagnosis. Moreover, the toxic effect of high concentration of serum bile acid was the main cause of perinatal adverse outcome and sudden death. However, the deficiency of this study is that the sample size is small, and the selection of cases is subjective to some extent. Therefore, the sample size should be expanded for further study in the later stage. In conclusion, this study provides a reference for the clinical diagnosis of ICP.

## Figures and Tables

**Figure 1:** Deep learning belief network model. (a) A stack of restricted Boltzmann machines; (b) corresponding deep learning belief network model.

**Figure 2:** Deep learning belief network model training process.

**Figure 3:** Error rate under different models. ∗Compared with DLBN, *P* < 0.05.

**Figure 4:** MRI manifestations of ICP pregnant women. (a) Patient 1, female, 35 years old, bile duct dilation with cholestasis in transverse position; (b) patient 1, female, 35 years old, with dilated bile ducts and coronal position with cholestasis; (c) patient 2, female, 29 years old, undilated bile duct with cholestasis in transverse position; (d) patient 2, female, 29 years old, coronal position with undilated bile duct and cholestasis.

**Figure 5:** Ten types of serum bile acid profile analysis. ∗Compared with the blank group, *P* < 0.05.

**Figure 6:** serum bile acid profile PLS-DA analysis results. (a) Experimental group serum bile acid profile PLS-DA two-dimensional score chart; (b) blank group serum bile acid profile PLS-DA three-dimensional score chart; and (c) histogram of the contribution value of ten different bile acids. The red represented the gallstone group, and blue represented the experimental group.

**Figure 7:** Serum bile acid profile PLS-DA analysis results of experimental group and gallstone group. (a) Experimental group serum bile acid profile PLS-DA two-dimensional score chart; (b) serum bile acid profile PLS-DA three-dimensional score chart of gallstone group; (c) histogram of the contribution value of 10 different bile acids. The green represented the gallstone group, and the yellow represented the experimental group.

**Figure 8:** Comparison results of the blood biochemical index levels of pregnant women in the experimental group and the blank group. (a) Comparison of TBA, TBIL, and DBIL levels; (b) comparison of ALT and AST levels. ∗Compared with the blank group, *P* < 0.05.

**Figure 9:** Expression of cord blood indicators in perinatal infants. (a) Comparison of serum biochemical indicators TBA; (b) comparison of myocardial enzyme spectrum CK and LDH; (c) cTnI comparison. ∗Compared with the blank group, *P* < 0.05.

**Figure 10:** Comparison of perinatal outcomes between the experimental group and the blank group. ∗Compared with the experimental group, *P* < 0.05.

## Data Availability

The data used to support the findings of this study are available from the corresponding author upon request.
